The article "An Efficient Cancer Classification Model Using Microarray and High-Dimensional Data" was published in 2021. Journal: Comput Intell Neurosci.

# An Efficient Cancer Classification Model Using Microarray and High-Dimensional Data

**DOI:** 10.1155/2021/7231126

**Published:** 2021-12-29

**Authors:** Hanaa Fathi, Hussain AlSalman, Abdu Gumaei, Ibrahim I. M. Manhrawy, Abdelazim G. Hussien, Passent El-Kafrawy

**Affiliations:** ^1^Mathematics and Computer Science Department, Faculty of Science, Menoufia University, Al Minufya, Egypt; ^2^Department of Computer Science, College of Computer and Information Sciences, King Saud University, Riyadh 11543, Saudi Arabia; ^3^Computer Science Department, Faculty of Applied Science, Taiz University, Taiz, Yemen; ^4^Department of Basic Science, Modern Academy, Cairo, Egypt; ^5^Department of Computer and Information Science, Linköping University, Linköping, Sweden; ^6^Faculty of Science, Fayoum University, Faiyum, Egypt; ^7^School of Information Technology and Computer Science, Nile University, Giza, Egypt

## Abstract

Cancer can be considered as one of the leading causes of death widely. One of the most effective tools to be able to handle cancer diagnosis, prognosis, and treatment is by using expression profiling technique which is based on microarray gene. For each data point (sample), gene data expression usually receives tens of thousands of genes. As a result, this data is large-scale, high-dimensional, and highly redundant. The classification of gene expression profiles is considered to be a (NP)-Hard problem. Feature (gene) selection is one of the most effective methods to handle this problem. A hybrid cancer classification approach is presented in this paper, and several machine learning techniques were used in the hybrid model: Pearson's correlation coefficient as a correlation-based feature selector and reducer, a Decision Tree classifier that is easy to interpret and does not require a parameter, and Grid Search CV (cross-validation) to optimize the maximum depth hyperparameter. Seven standard microarray cancer datasets are used to evaluate our model. To identify which features are the most informative and relative using the proposed model, various performance measurements are employed, including classification accuracy, specificity, sensitivity, *F*1-score, and AUC. The suggested strategy greatly decreases the number of genes required for classification, selects the most informative features, and increases classification accuracy, according to the results.

## 1. Introduction

Cancer can be considered as one of the leading death causes [1], and gene expression profiles derived from microarray data have been identified as promising cancer diagnostic indices [2].

Microarrays are used to measure thousands of genes interactions at the same time and create a cellular function global picture [3, 4].

The classification of microarray data is one of the most common and important applications of functional genomics microarray data which means classifying patients samples to many classes based on their gene expression profiles [5, 48]. In literature, there are many machine learning methods which have been used in the application of microarray data classification [7, 8]. However, the classification process of microarray data is still challenging and difficult due to the small samples numbers and its high dimensionality [9]. Microarray gene expression experiments often generate a lot of features for a small patients number which leads to a high-dimension dataset with a small samples number. Gene expression data is very challenging and complex; genes are correlated with one another directly or indirectly which make classification process a very hard and difficult mission which generally requires using an accurate and powerful feature selection technique.

The main phase in categorization systems is feature selection. To improve classification performance, feature selection-based classification approaches have been investigated. Any statistical technique's [10] success is contingent on the predetermination of independent properties. As a result, identification is kept to a minimum, but the purpose of feature selection is to find the most informative subset of characteristics and/or reduce the number of dimensions.

In order to be able to select an informative genes subset while eliminating/declining redundant or irrelevant genes and to be able to improve the performance of microarray high-dimension data classification, this research study introduces a hybrid feature selection approach, called PCC-DTCV, which combines different methods, Pearson's correlation coefficients (PCC) and Decision Tree (DT) [11] as classification approach and feature selection [12–17] and Grid Search CV which can be employed as an optimization technique [13, 14, 18–20, 42–47], to optimize the tuning parameters of DT (max-depth) to be able to get the optimal feature subset.

In order to evaluate the suggested PCC-DTCV model, 7 popular datasets from the most well-known used microarray datasets for different cancer types are used. The proposed model evaluation was carried out using classification accuracy, k-fold cross-validation, sensitivity, and specificity values.

The proposed method, according to the experimental methods, reduces dimensionality and selects the most important and informative features (genes) and improves the identification of cancer tissues from benign tissues. Furthermore, PCC-DTCV improves the accuracy classification performance.

## 2. Background and Related Work

Recently, there have been several major research efforts to study the classification and diagnosis of cancer microarray data. As a framework for the study presented in the remainder of the article, we offer an outline of some of this analysis and the applied techniques in Table 1.

## 3. Preliminaries

### 3.1. DNA Microarray

One of the main tools employed in molecular biology and genetics to track gene expression is the DNA microarray, which refers to the degree of development of genome-determined protein molecules. Although the protein structure varies from the mRNA measurement gene instead of protein structure, it is a popular method for calculating gene expression, so thousands of proteins would be difficult to analyse, and mRNA sequences [39] are hybridized with their additional DNA or RNA sequences, although proteins do not have these properties.  Figure 1 shows experimental microarray steps that include the extraction of mRNA from a cell or tissue. The structure of the DNA microarray matrix is shown in Figure 2, described by *N* (gene measurement) × *M* (a sample or condition involved in a specific microarray experiment).

The data on gene expression given by microarray experiments are processed as the broad matrix, where the samples are defined by the columns *S*{*S*_1_,…, *S*_*m*_} and *x*_*ij*_ measured the expression strength of the *i*-th gene (*i*=1,…, *n*, and *n* is the genes number) in the *j*-th sample (*j*=1,…, *m* and *m* characterize the  samples or experimental conditions). The row of genes represents *G* (gene_1_,…, gene_*n*_). In this study, we concentrate on solving two problems: the analysis and understanding of microarray data which have faced several challenges:

1. High dimensionality and noise
2. Increasing the accuracy performance taking into consideration interpretations that are biologically significant in gene expression when analysing microarray data

### 3.2. Decision Tree (DT)

Decision Tree learning can be considered as one of the most practical and commonly used methods for inductive inference.

It is a technique used for approximating discrete-valued functions that can learn disjunctive expressions and is resilient to noisy data [21]. These inductive inference algorithms are among the most common, and they have been successfully employed for a wide range of tasks, from learning up to diagnosis of the medical cases to learn to assess the loan applicants credit risk. Decision Tree learning is a nonbacktracking, one-step lookahead (hill-climbing) quest through the space of all possible Decision Trees using a heuristic. Decision Trees are commonly used in bioinformatics, especially in decision analysis to help identify a type of disease that is more likely to produce a specific symptom. A tree-based classifier was used in our proposed model PCC-DTCV for its basic properties, explicit context, and fast transformation to if-then law. The Decision Tree is a device for decision support which uses a dendritic graph and its potential problems, including unintended incident effects, resource costs, and utility. In bioinformatics, Decision Trees are widely used, especially in decision analysis to help classify a type of disease more likely to achieve a certain symptom. As a descriptive means for manipulating conditional probabilities, the Decision Tree may be used. This works to isolate and conquer [22] methods for creating a Decision Tree. As shown in equations (1)–(5), Entropy controls how a Decision Tree determines to divide the data. It influences how the borders are drawn by a Decision Tree. The Gini (Gini impurity) index measures the degree of probability of a feature that is incorrectly labelled to be randomly selected. The mistakes are in classification. The gain ratio is the parameter of the Decision Tree for measuring output and it is defined as

(1) $$\begin{array}{c} \text{Entropy }\left(\text{t}\right)=-\sum_{i=1}^{n}P\left(i|t\right){\text{log}}_{2}\;P\left(i|t\right), \end{array}$$

(2) $$\begin{array}{c} \mathrm{Gini}\left(t\right)=1-\sum_{i=1}^{n}{\left[P\left(i|t\right)\right]}^{2}, \end{array}$$

(3) $$\begin{array}{c} \text{Classification error}\left(t\right)=\;1\;-\max i\left[p\left(i|t\right)\right], \end{array}$$

where *n* is the number of classes and 0 log_20 = 0 in entropy calculations:

(4) $$\begin{array}{c} \mathrm{Gain Ratio}\;=\;\frac{\mathrm{Gain}\left(p\right)}{\mathrm{SplitInfo}\left(P\right)}, \end{array}$$

and the function SplitInfo is defined as follows:

(5) $$\begin{array}{c} \;\mathrm{Split}\;\mathrm{Info}\left(P\mathrm{,test}\right)=\sum_{i=1}^{n}P\left(\frac{i}{p}\right)\log\left(P\left(\frac{i}{p}\right)\right), \end{array}$$

where *p* gives the probability distribution of the data sample and “bit” due to calculating statistics. Equation (5) is used with log function with basis 2. The relation between Entropy, misclassification error, and Gini impurity is seen in Figure 3.

### 3.3. Correlation Coefficients

The Correlation-based Feature Selection algorithm computes the correlation coefficient using a correlation-based heuristic evaluation function (CFS). It gets over the limitation of univariate filter approaches which do not take into account feature interaction [23, 24]. The process of correlation [25] can be used to measure the relationship between variables (genes). The linear relationship between 2 variables can be described using Pearson's correlation coefficients or correlation coefficients in statistics. The well-known similarity measure between two features is defined as correlation. If two features depend on each other linearly then their coefficient of correlation is ±1. The correlation coefficient is 0 if the features are uncorrelated. For a pair of variables (*X*, *Y*), the coefficient of linear correlation *r* is given by the following equation [26]:

(6) $$\begin{array}{c} r=\frac{\sum \left(X_{i}-{\bar{X}}_{i}\right)\left(Y_{i}-{\bar{Y}}_{i}\right)}{\sqrt{\sum {\left(X_{i}-{\bar{X}}_{i}\right)}^{2}}\sqrt{\sum {\left(Y_{i}-{\bar{Y}}_{i}\right)}^{2}}}. \end{array}$$

In our model, we used Pearson's correlation coefficient (PCC) as feature selection [38]. This is a mathematical strength measure of a paired data linear relationship. It is defined by *r* and is limited as follows:

$\begin{array}{c} -1\leq r\leq 1 \end{array}$ , in which positive values mean that the linear correlation is positive, negative values imply that the linear correlation is negative, zero value means there is a nonlinear correlation, and the closer the value is to −1 or 1, the stronger the linear correlation exists.

The proposed model used Pearson's correlation to calculate the correlation between the features. Also using symmetric uncertainty measures, the class feature is calculated. If the value is higher than the threshold value (0.5), then the feature will be chosen. The selection ends when the number of features equals *n* log *n*. According to the decreasing order, each selected feature is ranked. To remove the redundant feature, the feature-feature correlation is done. Threshold values (0.4, 0.5, and 0.6) were used and their results were compared with the Decision Tree before and after the optimization of its maximum depth (max-depth).

### 3.4. Grid Search Cross-Validation

A Grid Search is a parameter tuning method which builds and evaluates a model methodically for each algorithm parameters combination specified in a grid. The well-known terms that should be addressed while using Grid Search CV are discussed as follows [27].

- *Estimator*. This term is used in order to implement the estimator interface in scikit-learn. This parameter receives the classifier to be trained [28].
- *Parameter Grid*. It is a Python key-value dictionary with pairs of parameter names and parameter settings. All combinations of these parameters are tested to ensure the highest level of accuracy.
- *Cross-Validation*. This determines the strategy for cross-validation splitting. Cross-validation is a technique to resample available data to evaluate machine learning models. The main goal of this is to evaluate the performance of machine learning models on previously unseen data. The main advantage of using this is that it produces less biased or optimistic results compared to a simple train-test split. The way it works is that it first shuffles the dataset randomly. The entire dataset is then divided into *k* groups. Each group is used as test data, while the others are used as training data. The evaluation band related to each group is saved to be summarized at the end to be able to check the performance of the model. Importantly, each sample appears once in the testing data and is used to train *k* − 1 times.  Figure 4 explains the Grid Search cross-validation process in detail.
- During the training step, hyperparameters that are optimizer variables are executed to get optimal average values after several trial-and-error processes. The tree maximum depth (max-depth) is the most critical hyperparameter that influences the difficulty of the Decision Tree model [6], whereas the maximum depth is the length of the longest distance from the tree root to a node. The root node is 0.0 in depth. The higher overall depth value induces overfitting, and the lower value results in underfitting. In the proposed hybrid model PCC-DTCV, Grid Search cross-validation is used to overcome the overfitting constraint with the regular Grid Search. To obtain better parameters, Grid Search cross-validation is used to optimize the tree maximum depth hyperparameter to get optimal hyperparameter value.

## 4. Proposed Model PCC-DTCV

The proposed hybrid model PCC-DTCV for classifying and diagnosing cancer microarray data (as shown in Figure 5) will be clarified in detail. Key model phases are as follows: (1) The datasets (cancer microarray) are preprocessed. This stage is essential to (a) avoid features in wide digital ranges dominating fewer ranges, (b) avoid numeric complexities through calculation, and (c) adjust each feature to the range [0,1]. (2) PCC is applied for finding the association between the continuous features and the class feature, evaluation to genes is based on how it is related to targeting the features that have a high correlation with the target class having a correlation value near to 1, and the genes with the correlation coefficient ≥0.5 are removed and the output subsets are informative and important genes (features). (3) The sample data output subset is the partition used to train data to match the model and test data used to validate the model as soon as a model is fully trained (trained DT). (4) Grid Search CV with 10-fold cross-validation is used to obtain the optimal parameters (max-depth) of the tree on the training set. (5) Model accuracy is evaluated, using 10-fold cross-validation, and our dataset is 10-fold split, using train split to train the classifier, and prediction quality on unseen data is estimated (test split). The confusion matrix is measured for test split. The AUC, specificity, and sensitivity in addition to accuracy are computed. (6) If the termination conditions are not met, the process from three to six is repeated until the termination criteria are satisfied. If the termination is fulfilled (max folds, number = 10), the result will be a subset of optimal genes (features) with the most important and informative genes.

## 5. Results and Discussion

In the following section, the findings of numerous studies that have been performed to determine the efficacy of the proposed hybrid model PCC-DTCV are discussed. A PC with the following properties is the platform used to test the proposed model: RAM 4 GB and 32-bit OS (Windows 7), Intel(R) Core (TM) i5-7500CPU, as well as frameworks such as Pandas, NumPy, Keras, SciPy, and Matplotlib and the Python programming language. The datasets for human cancer research included the following: breast cancer, prostate, colon tumor, lung cancer, and leukemia were applied to 7 different microarray datasets with a limited sample and high-dimensional and binary class. Also, all datasets have two types, and Table 2 lists the definitions of all datasets.

In all studies, 10-fold cross-validation techniques were applied. The data were randomly divided into 10 different subsets (with the same size in 10-fold cross-validation), and the experiment was conducted 10 times. One subset was used as a test set for each run, and one was used as a validation set, and the other sets were used as a training set (Figure 5). To obtain a single estimate, the mean of the *k* results from the folds can then be determined. To approximate the model, 10-fold cross-validation was used in our experiments, and the results obtained are illustrated in the form of mean ± standard deviation. Also, in both analyses, the number of iterations was 50. The value of the tree (max-depth) hyperparameter is [3, 30]. Our evaluation included the four following measurements:

1. Accuracy (ACC): it is the most used evaluation standard for the proportion of correctly predicted pairs, but using it alone is usually insufficient. Accuracy (ACC)=((TP+TN)/(TP+TN+FP+FN)).
2. Sensitivity (Sen.): a diseased person is likely to be recognized as diseased through the test. *S*=(TP/(TP+TN)), where TN is the true negatives number and TP is the true positives number.
3. Specificity (Spec.): the likelihood is that a person without the illness is defined by the test as nondiseased (or healthy). It is described as TRN=(TN/(TP+TN)), where FP implies the number of false positives and TN is the number of true negatives.
4. The AUC shows the area under the receiver operating characteristics (ROC) curve, and it is calculated as AUC=(1+TPR − FPR)/2.

TP is true positive, FP is false positive, TN is true negative, and FN is false negative. Based on the confusion matrix, we evaluated the performance of the proposed method and rival gene selection. To assess the output of our model, a statistical test method called Chi-Square test [21] is used to check how well the observed values for a given distribution fit the distribution when the variables are independent.

## 6. Experimental Results

The experimental results are discussed in this section to validate the performance of the our model PCC-DTCV. The classification accuracy performance and the selected feature (genes) numbers of the PCC-DTCV method with PCC (0.4, 0.5, and 0.6) for all microarray datasets, respectively, are summarized in Tables 3–8 and Figures 6–9. The statistical model is described in Table 9. Six different performance metrics were chosen for result estimation: AUC, ACC, specificity, sensitivity, recall, and *F*1-score [10, 22]. To reduce the high dimensionality, improve the classification performance of the problem at hand, and select the most informative genes, we run PCC-DTCV using all datasets and get the informative selected features (genes) number. It can be noted that PCC-DTCV gives the genes (features) ordered list according to the highest correlation informative, importance, and relevant genes. It is obvious that PCC-DTCV achieves the highest level of dimensional reduction by choosing smallest number of informative genes and the biggest dimensional dataset is Chowdary for breast cancer with 22283 features (genes) and 104 samples, as seen in Tables 3 and 4. The highly correlated subset selected genes with the target class by the PCC-DTCV with PPC ≥= 0.4 are 410 features (genes) from 22283. PCC-DTCV compared the performance of DT classifier without any optimization method and optimized DT as given in Tables 3 and 4, respectively, as well as the accuracy of the highest-dimensional dataset with PPC ≥= 0.4 with optimized DT classifier and DT classifier. With accuracy of (0.92 ± 0.09), the optimized DT classifier shows better accuracy than DT classifier with accuracy of (0.90 ± 0.09).

Tables 5 and 6 show that the number of selected (features) genes with PPC ≥0.5 is lower than the number of selected (features) genes with PPC ≥0.4 for all datasets; it means that the PCC-DTCV achieved higher-dimensional reduction with PPC ≥0.5 than with PPC ≥0.4. In terms of ACC, AUC, sensitivity, and specificity, the PCC-DTCV achieved higher results compared to those achieved with PPC ≥0.4 with both optimized DT classifier and DT classifier; for example, the number of selected (features) genes of Gordon dataset for lung cancer is 274 compared with 743 for PPC ≥0.4, in addition to the values of 94%, 88%, 97%, and 79% for terms ACC, AUC, sensitivity, and specificity with DT classifier and 94%, 90%, 97%, and 87% with optimized DT classifier. From Tables 7 and 8, we can see that the PCC-DTCV with PPC ≥0.6 has the best ACC, AUC, sensitivity, specificity, recall, and *F*1-score compared to PPC ≥0.4 and 0.5, which means that the classification performance of PCC-DTCV is best with PPC ≥0.6 and the selected genes (features) are the most relevant, important, and informative genes.

Figures 6–9 represent the classification performance obtained using PPC ≥0.4, 0.5, and 0.6 and DT classifier with the PCC-DTCV model for prostate cancer, colon cancer, leukemia, lung cancer, and breast cancer datasets. From Figure 6, the achieved results show that the suggested PCC-DTCV model gives better accuracy for breast cancer, lung cancer, and leukemia datasets and can obtain the highest accuracy with PPC ≥0.6 in the Chowdary dataset for breast cancer, 96%. From Figure 7, the AUC metric obtains more than 90% for both Chowdary and Singh datasets and more than 80% for all datasets except Alon dataset for colon cancer, obtaining 71% for PPC ≥0.6. From Figure 8, the sensitivity metric obtains more than 90 with Gordon, Chowdary, and Golub datasets for lung cancer, breast cancer, and Leukemia, respectively, with PPC ≥0.4, 0.5, and 0.6. Specificity metric shown in Figure 9 achieves 96% for Chowdary dataset with PPC ≥0.6.

Figures 10–13 represent the classification performance obtained using optimized DT classifier and PPC with PCC-DTCV model for prostate cancer, colon cancer, leukemia, lung cancer, and breast cancer datasets. In Figure 10, accuracy metric can obtain more than 90% for Gordon, Chowdary, and Golub datasets for lung cancer, breast cancer, and leukemia, respectively, with PPC ≥0.6. From Figure 11, the AUC metric obtains more than 80% for all datasets except Alon dataset for colon cancer, obtaining 76% for PPC ≥0.6. From Figure 12, the sensitivity metric obtains more than 90% with Gordon, Chowdary, and Golub datasets for lung cancer, breast cancer, and leukemia, respectively, with PPC ≥0.4, 0.5, and 0.6. Specificity metric shown in Figure 13 obtains more than 80% for all datasets with PPC ≥ 0.6. Finally, the proposed model gives the best classification performance with PPC ≥0.6 for both optimized DT classifier and DT classifier and the selected features (genes) have minimum redundancy and are maximally relevant and informative with high correlation with target class.

These results clarify that the proposed models follow a normal distribution as the value in both Kolmogorov–Smirnov and Shapiro–Wilk Sig. 0.02 ≥ .05 shown in Table 9. The first condition is fulfilled by following a normal distribution. The second condition is that there are no outliers and anomalies, as well as applying regression analysis to use the Manhattan distance method, which calculates the outlier values. In addition, the emergence of a new variable and the largest value in Manhattan distance is compared and it is less valuable than the number of existing variables using the Chi-Square. The value of Manhattan distance = 18.466 compared to using the Chi-Square. The critical value of the Chi-Square distribution will be applied at d*f* = 6 and the *p* value of 0.001 is found to be at 0.999 confidence interval and uncertainty interval 0.001. If the value of 22.46 is greater than 18.466, then it is assumed that there are no multiple-choice outliers. Sig = .0155, which is greater than 0.0001. It is a fulfilled condition and it means that the homogeneity condition variance exists and is fulfilled by a choice of Finney greater than 0.5. This indicates that the variance of the dependent variables is equal.

## 7. Conclusions

This paper presents a PCC-DTCV model for cancer diagnosis and classification. PCC-DTCV optimizes the tuning parameter (max-depth) of the DT classifier using Grid Search and Pearson's correlation used as a gene (feature) selection method. The proposed model was effective in identifying an optimal or near-optimal subset of informative and important genes and yielded high classification results. Several experiments were carried out to evaluate the proposed PCC-DTCV model for selecting the most informative genes to improve the performance classification of cancer microarray data. In addition to reducing the dimensionality of microarray data, the result demonstrates the model's effective performance in selecting the most informative genes with high importance. The results showed that PCC-DTCV provides the best fit for cancer type prediction in terms of specificity, AUC, sensitivity, and accuracy. In future work, for Decision Tree optimization, we anticipate using ski driver and other algorithms.

## Figures and Tables

**Figure 1:** Experiment steps of microarray.

**Figure 2:** Microarray data matrix structure.

**Figure 3:** The relation between Gini impurity, Entropy, and misclassification error. [22].

**Figure 4:** Working of Grid Search cross-validation [26].

**Figure 5:** Proposed model (PCC-DTCV).

**Figure 6:** Accuracy obtained for PCC-DTCV model using the DT classifier with PPC ≥0.4, 0.5, and 0.6 for all datasets.

**Figure 7:** AUC obtained for PCC-DTCV model using the DT classifier with PPC ≥0.4, 0.5, and 0.6 for all datasets.

**Figure 8:** Sensitivity obtained for PCC-DTCV model using the DT classifier with PPC ≥0.4, 0.5, and 0.6 for all datasets.

**Figure 9:** Specificity obtained for PCC-DTCV model using the DT classifier with PPC ≥0.4, 0.5, and 6 for all datasets.

**Figure 10:** Accuracy obtained for PCC-DTCV model using the DT classifier with PPC ≥0.4, 0.5, and 0.6 for all datasets.

**Figure 11:** AUC obtained for PCC-DTCV model using the DT classifier with PPC ≥0.4, 0.5, and 0.6 for all datasets.

**Figure 12:** Sensitivity obtained for PCC-DTCV model using the optimized DT classifier with PPC ≥0.4, 0.5, and 0.6 for all datasets.

**Figure 13:** Specificity obtained for PCC-DTCV model using the optimized DT classifier with PPC ≥0.4, 0.5, and 0.6 for all datasets.

**Table 1:** Review of previous studies on the feature selection, optimization, and classification methods.

Author	Datasets	Method	Remark
[29] Shukla and Tripathi (2020)	DLBCL	(JMI) Joint mutual information (mRMR) information gain (IG)	This research introduced modern filter-based gene selection technique for detecting biomarkers from microarray data.
[30] Kilicarslan et al. (2020)	Ovarian, leukemia, and Central Nervous system (CNS)	Relief-F of support vector machines (SVM), coevolutionary neural networks (CNN)	This research introduced a hybrid approach based on Relief-F and CNN for cancer diagnosis and classification.
[31] Pashaei et al. (2016)	Colon tumor ALL, AML, 4 (CNS) MLL	Binary black hole algorithm (BBHA) and random forest ranking (RFR)	The authors introduced gene selection and classification techniques to microarray data based on RFR and BBHA.
[32] Pradana and Aditsania	Breast cancer	Binary particle swarm optimization (BPSO) and Decision Tree C4.5	This research introduced binary PSO and DT for cancer detection based on microarray data classification.
[33] Mantovani et al.	UCI	J48 DTs	They presented induction algorithm and introduced hyperparameter tuning of a Decision Tree induction algorithm.
[34] Abbas et al. (2021)	Breast cancer	Whale optimization algorithm (WOA), extremely randomized tree BCD-WERT	This research introduced a novel model for breast cancer detection using WOA optimization based on extremely randomized tree algorithm and efficient features.
[35] Reddy et al.	Srivastava, G. (2020)	UCI heart disease	This research presented an adaptive genetic fuzzy logic algorithm and introduced a hybrid GA and a fuzzy logic classifier for heart diagnosis and disease.
[36] Qaraad et al. (2020)	Colon cancer, breast cancer, prostate cancer	Elastic NET PSO algorithm	This research introduced parameters optimization of Elastic NET using PSO algorithm for high-dimensional data.
[37] El Kafrawy et al. (2020)	De novo acute myeloid leukemia	Recursive feature elimination (RFE), tree-based feature selection (TBFS)	This research introduced multifeature selection with machine learning for de novo acute myeloid leukemia in Egypt.
[38] Turgut et al. (2020)	Breast cancer	AdaBoost and Gradient Boosting random forest, logistic regression	This research introduced classification for microarray breast cancer data using machine learning methods.

**Table 2:** Characterization of the dataset.

Disease	Dataset	No. of samples	No. of features
Prostate cancer	D1, Singh [21]	102	12600
Lung cancer	D2, Gordon [22]	181	12533
Breast cancer	D3, Chowdary [23]	104	22283
Colon cancer	D4, Alon [24]	62	2000
Breast cancer	D5, Chin [25]	118	22215
Breast cancer	D6, West [26]	49	7129
Leukemia	D7, Golub [27]	72	7129

**Table 3:** PCC-DTCV model with DT and PPC ≥0.4.

Dataset	Features	Selected features	PCC-DTCV model with DT and PPC ≥0.5							
			Accuracy	AUC	Sensitivity	Specificity	Recall		*F*1-score	
							0	1	0	1
Singh	12600	299	0.77 ± 0.16	0.78 ± 0.16	0.78 ± 0.19	0.77 ± 0.20	0.80	0.79	0.79	0.80
Gordon	12533	743	0.93 ± 0.06	0.88 ± 0.11	0.97 ± 0.06	0.79 ± 0.24	0.95	0.71	0.95	0.73
Chowdary	22283	410	0.90 ± 0.09	0.89 ± 0.08	0.90 ± 0.15	0.88 ± 0.12	0.94	0.88	0.93	0.89
Alon	2000	61	0.79 ± 0.20	0.075 ± 0.22	0.62 ± 0.37	0.88 ± 0.20	0.64	0.82	0.65	0.81
Chin	22215	1211	0.81 ± 0.12	0.80 ± 0.11	0.78 ± 0.13	0.82 ± 0.17	0.79	0.85	0.77	0.86
West	7129	28	0.83 ± 0.15	0.84 ± 0.16	0.82 ± 0.23	0.87 ± 0.16	0.84	0.83	0.84	0.83
Golub	7129	465	0.89 ± 0.11	0.87 ± 0.13	0.93 ± 0.10	0.80 ± 0.21	0.89	0.76	0.88	0.78

**Table 4:** PCC-DTCV model with optimized DT and PPC ≥0.4.

Dataset	Features	Selected features	PCC-DTCV model with optimized DT and PPC ≥0.5							
			Accuracy	AUC	Sensitivity	Specificity	Recall		*F*1-score	
							0	1	0	1
Singh	12600	299	0.76 ± 0.12	0.76 ± 0.12	0.74 ± 0.16	0.78 ± 0.21	0.80	0.81	0.80	0.81
Gordon	12533	743	0.93 ± 0.05	0.87 ± 0.11	0.97 ± 0.04	0.76 ± 0.23	0.97	0.84	0.97	0.84
Chowdary	22283	410	0.92 ± 0.09	0.92 ± 0.09	0.94 ± 0.12	0.90 ± 0.12	0.94	0.88	0.93	0.83
Alon	2000	61	0.82 ± 0.13	0.80 ± 0.14	0.73 ± 0.23	0.88 ± 0.17	0.73	0.82	0.71	0.84
Chin	22215	1211	0.79 ± 0.09	0.78 ± 0.10	0.74 ± 0.17	0.81 ± 0.12	0.72	0.85	0.73	0.85
West	7129	28	0.86 ± 0.13	0.87 ± 0.13	0.87 ± 0.21	0.87 ± 0.16	0.84	0.83	0.84	0.83
Golub	7129	465	0.86 ± 0.09	0.83 ± 0.12	0.92 ± 0.10	0.75 ± 0.21	0.94	0.80	0.92	0.83

**Table 5:** PCC-DTCV model with DT and PPC ≥0.5.

Dataset	Features	Selected features	PCC-DTCV model with optimized DT and PPC ≥0.5							
			Accuracy	AUC	Sensitivity	Specificity	Recall		*F*1-score	
							0	1	0	1
Singh	12600	58	0.82 ± 0.11	0.82 ± 0.10	0.88 ± 0.13	0.77 ± 0.20	0.88	0.77	0.83	0.82
Gordon	12533	274	0.94 ± 0.05	0.88 ± 0.11	0.97 ± 0.05	0.79 ± 0.24	0.97	0.81	0.97	0.83
Chowdary	22283	39	0.91 ± 0.15	0.90 ± 0.15	0.94 ± 0.12	0.86 ± 0.19	0.95	0.90	0.94	0.92
Alon	2000	9	0.73 ± 0.18	0.70 ± 0.17	0.63 ± 0.24	0.78 ± 0.21	0.59	0.80	0.60	0.79
Chin	22215	305	0.81 ± 0.09	0.80 ± 0.08	0.75 ± 0.10	0.85 ± 0.14	0.72	0.85	0.73	0.85
West	7129	5	0.90 ± 0.13	0.91 ± 0.13	0.92 ± 0.17	0.90 ± 0.15	0.92	0.88	0.83	0.82
Golub	7129	133	0.87 ± 0.08	0.85 ± 0.10	0.94 ± 0.09	0.77 ± 0.20	0.91	0.80	0.91	0.82

**Table 6:** PCC-DTCV model with optimized DT and PPC ≥0.5.

Dataset	Features	Selected features	PCC-DTCV model with optimized DT and PPC ≥0.5							
			Accuracy	AUC	Sensitivity	Specificity	Recall		*F*1-score	
							0	1	0	1
Singh	12600	58	0.78 ± 0.15	0.78 ± 0.15	0.78 ± 0.19	0.78 ± 0.23	0.78	0.83	0.80	0.81
Gordon	12533	274	0.94 ± 0.04	0.90 ± 0.08	0.97 ± 0.04	0.84 ± 0.16	0.95	0.77	0.95	0.77
Chowdary	22283	39	0.94 ± 0.08	0.94 ± 0.08	0.95 ± 0.09	0.93 ± 0.11	0.95	0.90	0.94	0.92
Alon	2000	9	0.78 ± 0.19	0.75 ± 0.19	0.68 ± 0.26	0.82 ± 0.23	0.68	0.80	0.67	0.81
Chin	22215	305	0.82 ± 0.09	0.80 ± 0.09	0.77 ± 0.15	0.84 ± 0.12	0.74	0.85	0.74	0.85
West	7129	5	0.83 ± 0.18	0.83 ± 0.18	0.80 ± 0.24	0.87 ± 0.16	0.84	0.83	0.84	0.83
Golub	7129	133	0.89 ± 0.06	0.89 ± 0.07	0.92 ± 0.10	0.85 ± 0.19	0.87	0.76	0.87	0.76

**Table 7:** PCC-DTCV model with DT and PPC ≥0.5.

Dataset	Features	Selected features	PCC-DTCV model with optimized DT and PPC ≥0.5							
			Accuracy	AUC	Sensitivity	Specificity	Recall		*F*1-score	
							0	1	0	1
Singh	12600	10	0.90 ± 0.08	0.90 ± 0.08	0.90 ± 0.10	0.90 ± 0.10	0.90	0.88	0.89	0.89
Gordon	12533	98	0.95 ± 0.05	0.89 ± 0.11	0.98 ± 0.04	0.81 ± 0.22	0.99	0.74	0.97	0.84
Chowdary	22283	5	0.96 ± 0.06	0.96 ± 0.06	0.97 ± 0.06	0.96 ± 0.12	0.95	0.93	0.95	0.93
Alon	2000	1	0.72 ± 0.18	0.71 ± 0.19	0.67 ± 0.32	0.75 ± 0.22	0.68	0.75	0.64	0.78
Chin	22215	54	0.85 ± 0.07	0.84 ± 0.08	0.82 ± 0.17	0.87 ± 0.11	0.72	0.88	0.75	0.86
West	7129	2	0.82 ± 0.19	0.82 ± 0.21	0.87 ± 0.32	0.85 ± 0.19	0.80	0.83	0.82	0.82
Golub	7129	36	0.85 ± 0.10	0.82 ± 0.12	0.89 ± 0.11	0.75 ± 0.21	0.94	0.80	0.92	0.83

**Table 8:** PCC-DTCV model with optimized DT and PPC ≥ 0.6.

Dataset	Features	Selected features	PCC-DTCV model with optimized DT and PPC ≥0.5							
			Accuracy	AUC	Sensitivity	Specificity	Recall		*F*1-score	
							0	1	0	1
Singh	12600	10	0.89 ± 0.05	0.89 ± 0.05	0.88 ± 0.10	0.90 ± 0.13	0.88	0.94	0.91	0.92
Gordon	12533	98	0.95 ± 0.04	0.87 ± 0.11	0.99 ± 0.03	0.75 ± 0.23	0.99	0.77	0.97	0.84
Chowdary	22283	5	0.93 ± 0.06	0.93 ± 0.07	0.95 ± 0.07	0.91 ± 0.14	0.97	0.90	0.95	0.93
Alon	2000	1	0.79 ± 0.18	0.76 ± 0.17	0.67 ± 0.22	0.85 ± 0.25	0.64	0.88	0.68	0.84
Chin	22215	54	0.84 ± 0.11	0.83 ± 0.12	0.78 ± 0.20	0.88 ± 0.09	0.79	0.83	0.76	0.85
West	7129	2	0.83 ± 0.15	0.83 ± 0.17	0.78 ± 0.32	0.88 ± 0.18	0.80	0.83	0.82	0.82
Golub	7129	36	0.90 ± 0.09	0.88 ± 0.12	0.96 ± 0.08	0.80 ± 0.21	0.91	0.80	0.91	0.80

**Table 9:** Tests of normality.

		Kolmogorov–Smirnov^a^		Shapiro−Wilk	
		PCR	Statistic	Sig.	Statistic
Spec. DT OPT	≥0.4	0.158	0.200^*∗*^	0.983	0.971
	≥0.5	0.166	0.200^*∗*^	0.943	0.668
	≥0.6	0.257	0.178	0.940	0.639

AUC DT OPT	≥0.4	0.161	0.200^*∗*^	0.981	0.965
	≥0.5	0.190	0.200^*∗*^	0.956	0.190
	≥0.6	0.205	0.200^*∗*^	0.892	0.285

Sen. DT OPT	≥0.4	0.137	0.200^*∗*^	0.962	0.832
	≥0.5	0.163	0.200^*∗*^	0.926	0.517
	≥0.6	0.245	0.200^*∗*^	0.884	0.245

Sen. DT	≥0.4	0.205	0.200^*∗*^	0.871	0.189
	≥0.5	0.241	0.200^*∗*^	0.873	0.197
	≥0.6	0.275	0.117	0.905	0.364

Spec. DT	≥0.4	0.284	0.093	0.836	0.090
	≥0.5	0.169	0.200^*∗*^	0.956	0.785
	≥0.6	0.188	0.200^*∗*^	0.911	0.403

AUC DT	≥0.4	0.204	0.200^*∗*^	0.948	0.714
	≥0.5	0.243	0.200^*∗*^	0.900	0.334
	≥0.6	0.233	0.200^*∗*^	0.933	0.580

^*∗*^This is a lower bound of the true significance. ^a^Lilliefors significance correction.

## Data Availability

The data used to support the findings of this study are available from the corresponding author upon request.
